# Research on the Intervention Countermeasures and Mental Health Status of College Music Teachers from the Perspective of Positive Psychology

**DOI:** 10.1155/2022/9133979

**Published:** 2022-02-28

**Authors:** Keshuang Liu

**Affiliations:** School of Music and Dance, ChangSha Normal University, ChangSha, Hunan 410000, China

## Abstract

The goal of education is to train people who are well-rounded and educate people with heart through teachers and determine the direction for the growth of life. Psychological education is one of the top ten education systems in colleges and universities. The psychological health of college teachers is the key to teaching and education. Colleges and universities attach great importance to teachers' educational level and scientific research achievements, pay attention to teachers' instrumental value, and pay little attention to teachers' mental health. Therefore, this study aims to study the mental health status and prevention measures of college music teachers from the perspective of positive psychology. By combining the qualitative method with the quantitative method, this study carries out questionnaire survey and interview on “mental health” of music teachers in four universities and then puts forward relevant intervention countermeasures. Research shows that only one-fifth of the teachers believed that they had received psychological counseling from the school and successfully solved their own problems; nearly 60% of music teachers said that the psychological counseling provided by the school lacked pertinence and professionalism, and lacked practical solutions to their own problems. This shows that the psychological intervention strategies adopted by Chinese colleges and universities for music teachers are far from the expected results.

## 1. Introduction

With the continuous development of China's economy, the reform of colleges and universities has entered the deep water zone, and higher education has received widespread attention. Teachers need to have higher academic qualifications and scientific research capabilities [1, 2]. College teachers are mental workers who are responsible for educational and teaching tasks and scientific research, which puts forward higher requirements for college teachers, so their psychological pressure is huge [3, 4].

At present, the enrollment expansion of colleges and universities is a general trend, and the scale of college students is increasing, but the number of university teachers does not match, which leads to the increasing teaching and scientific research tasks of university teachers [5, 6]. The burden from many aspects will inevitably reduce the teaching effect and enthusiasm and bring a certain negative impact on the work efficiency of teachers, so that teaching and scientific research cannot achieve the desired results, and the performance of colleges and universities will also be affected [7, 8].

As an important subject of quality education, music education has not received enough attention in colleges and universities. Although the work of most music teachers is relatively easy, there is neither teaching pressure nor many requirements for the development of teaching. But at the same time, many colleges and universities not only have insufficient protection for music teachers in terms of educational resources but also have great disadvantages in terms of professional title promotion. Most college music teachers have difficulty impressing their students. All these bring psychological pressure to college teachers. In addition, college music teachers are also facing pressure from family, society, and other aspects. The survey shows that more than 70% of music teachers in colleges and universities believe that they are suffering from job burnout, and 64.7% of teachers believe that their sense of professional achievement is too low. These indicate that the mental health of music teachers in colleges and universities in my country must be followed closely.

This study conducts a questionnaire survey and interviews on the “mental health” of music teachers in four universities through questionnaire surveys and then provides relevant intervention strategies. The results show that only 21% of teachers attach importance to mental health and have achieved good results; 58% of music teachers said that colleges and universities pay attention to it and take certain measures to alleviate the psychological pressure of college teachers, but for some reasons or because college music teachers do not participate and insist, the effect is not good.

## 2. Mental Health of Music Teachers in Colleges and Universities from the Perspective of Positive Psychology

### 2.1. Research Methods

This article chooses the questionnaire survey method, as well as a combination of qualitative and quantitative research methods. The questionnaire survey method makes the survey results easy to quantify and convenient for statistical analysis. Qualitative research and quantitative research can complement each other, strengthen each other, and make the results more accurate.

#### 2.1.1. Questionnaire Survey Method

The questionnaire survey method is based on the written form to obtain information, which is an indirect way of obtaining information. Send the enquiry form to the respondent, and the respondent fills it out according to the content of the form, seeking truth from facts. This questionnaire formed a preliminary questionnaire after conducting in-depth interviews with literature data sorting and referring to the maturity scale. So, a small-scale test was carried out and then revised and then formally distributed.

#### 2.1.2. The Method of Combining Qualitative Research and Quantitative Research

Through qualitative analysis, combined with the normative research method and empirical research method, this study makes the empirical research more objective, real, and comprehensive. On the basis of qualitative research, the scientific of the demonstration process can be effectively improved, and the persuasion of the result of the demonstration can be enhanced by quantitative research.

### 2.2. The Healthy Mental Performance of College Music Teachers from the Perspective of Positive Psychology

#### 2.2.1. Good Health

Physical and mental health is a prerequisite for teachers to work, and this depends on the following aspects. The first is quality sleep. Data show that at this stage, about 27.4% of music teachers in colleges and universities in my country have sleep disorders, which have a certain impact on their health [9, 10]. The second is to follow comprehensive and scientific diets. Music teachers in colleges belong to the middle and high income groups. This income level makes their diets continue to improve, and the number of teachers in the three high schools continues to grow. The third is to insist on physical exercise. College teachers with a good mental state will arrange proper physical exercise, strengthen limbs, and increase resistance and strong physical recovery ability while doing mental work [11, 12].

#### 2.2.2. High Self-Awareness

First, college teachers can be neither inferior nor conceited [13, 14]. Second, they can actively accept themselves be able to believe in themselves, forgive themselves, face up to themselves, and be willing to accept their appearance, shape, and personality characteristics. Finally, they can grasp their own expectations, understand and practice new roles, and have good adaptability to the changes in their environment.

#### 2.2.3. Optimistic, Strong Willpower

College teachers should use their own optimistic mental state to infect and drive the classroom atmosphere. Teaching and learning are interactive activities [15, 16]. Optimism of character is an important condition for music teachers to get rid of subjective and objective troubles and better devote themselves to work and life. Optimistic personality makes music teachers relax at work, and their performance in the classroom can more resonate with students and use their optimistic attitude to infect and drive the classroom atmosphere.

#### 2.2.4. Active Dedication and Strong Sense of Responsibility

The common desire of every college teacher is to let students fully grasp the knowledge they teach. For this goal, teachers can teach tirelessly, repeat continuously, and can also endure boring. These are the most active and dedicated teachers of colleges and universities. Good embodiment: the responsibility of college teachers is to impart knowledge, responsible for students' knowledge and national talent training.

### 2.3. Causes of Mental Health Problems

#### 2.3.1. Differences in Individual Psychological Quality of College Teachers

Individual psychological quality is the basis for teachers' externalizing state when faced with troubles in life and work. There are differences in psychological quality, which lead to the psychological problems of some college music teachers cannot be solved satisfactorily. After all, individual psychological quality is a very broad category, which includes many fields [17]. This requires us to seek truth from facts and formulate targeted strategies when actively intervening.

#### 2.3.2. College Teachers Lack the Ability of Self-Psychological Intervention

At this stage, college teachers in our country generally lack mature self-psychological intervention and adjustment ability. Active psychological intervention has only been introduced into my country's higher education in recent years. Music teachers have neither had professional theoretical training nor mature cases for reference [18, 19]. At the same time, many colleges and universities are still in the exploratory stage for the construction of teachers' psychological intervention system and have not formed a complete system yet [20, 21].

#### 2.3.3. Occupational Pressure of Teachers' Work

Colleges and universities have clearly defined the goals and directions of music teaching, but the actual teaching effect of each college is far from the expected. At present, although Chinese students have been exposed to music since primary school, most of them have little knowledge of music because of their long-term position as a “small subject.” Few of them would develop a strong interest in music, even at the university stage, when the academic pressure was the most relaxed. Under such a background, the teaching system of colleges and universities with music appreciation and music literacy as the training goal appears to be more high and low [22, 23]. As a result, although the work of music teachers in colleges and universities seems to be easy, in fact, the students they face have a very poor foundation in the field of music, which brings them considerable work pressure.

#### 2.3.4. Life Pressure of Family Emotions

The negative emotions formed by the pressure of college teachers at work will directly or indirectly affect the emotions of the family and relatives, and the negative emotions generated in the family and emotions will also affect the work of college teachers; that is, work factors make college teachers unable to fulfill their responsibilities to the family, and the burden of the family will also cause work. Interference affects the personal development of college teachers [24].

#### 2.3.5. Pressure from the Social Level

University teachers are leaders in the production and dissemination of knowledge and shoulder the important task of cultivating talents for the country. The society has relatively high requirements for college teachers, and every word and deed of college teachers is subject to the supervision of the masses. Therefore, college teachers are under tremendous pressure from the society.

## 3. Experiment

### 3.1. Research Purpose

The physical and mental health of college teachers has many aspects, which have a series of negative effects on the quality of life and work of teachers, and also affect the physical and mental health of college students. Education authorities are paying more and more attention to the mental health of this group, helping them to adjust their mentality through supporting reforms and active psychological intervention. Teachers are also paying more and more attention to personal health. However, after several years of hard work, the mental health of music teachers in colleges and universities is still in a worrying state.

### 3.2. Questionnaire Design

The subjects of this questionnaire are music teachers from four colleges and universities in Chengdu, Sichuan Province. The survey site is the music teacher teaching and research group offices of these four colleges and universities. The survey is randomly distributed and collected in due course. The questionnaire is in the form of selective answers. A total of 63 questionnaires were distributed. After collecting and sorting out statistics, 59 valid questionnaires were finally formed, with a recovery rate of over 90%, which can truly and effectively reflect the actual situation of the surveyed questions. After the questionnaire is recovered, after careful analysis and research, the questionnaire reflects the outstanding problems and anonymous visits to some college music teachers, in order to further obtain the psychological status and the main reasons for the psychological production of college teachers, and find out the solutions.

### 3.3. Algorithm

Correlation analysis usually refers to a real relationship between subjective and objective phenomena. However, in terms of quantity, it is not strictly dependent. There are two forms of correlation determination here: qualitative and quantitative analysis. Qualitative analysis is mainly based on the theoretical knowledge and practical experience of the researcher to determine whether there is a correlation between objective phenomena and what kind of relationship. This analysis method is subjective and relatively strong. Among them, the commonly used calculation formulae are

(1) $$\begin{array}{c} y=\frac{p^{2}ij}{p_{i}p_{j}}=\frac{\sum \left(i-i^{\prime }\right)\left(j-j^{\prime }\right)/m}{\sqrt{\sum {\left(i-i^{\prime }\right)}^{2}/m}\sqrt{\sum {\left(j-j^{\prime }\right)}^{2}/m}}, \end{array}$$

(2) $$\begin{array}{c} y=\frac{m\sum ij-\sum i\sum j}{\sqrt{m\sum i^{2}-{\left(\sum i\right)}^{2}}\sqrt{\sum j^{2}-{\left(\sum j\right)}^{2}}}. \end{array}$$

## 4. Discussion

### 4.1. Physical Health Problems and Emotional Conditions

It can be seen from Figure 1 that 16% of the music teachers surveyed often feel tired at work, decreased energy, memory decline, and prone to insomnia. Dat shows that college music teachers are troubled by this symptom. Chengdu is different; in terms of emotional state, 20% of music teachers often experience emotional fluctuating, annoying, and agitated states. These states will be in the work and life of music teachers, appeared in and caused a certain impact.

### 4.2. Sources of Stress

Table 1 provides the pressure of college music teachers on the current working environment. In terms of pressure sources, assessment, appraisal, scientific research, and promotion of professional titles are the main pressures in teachers' work; in life, the main pressure sources of college music teachers are financial burdens, interpersonal relationships, and children's education issues.

### 4.3. Mental Health Attention

In terms of the degree of college's attention to the mental health of teachers, as shown in Figure 2, the survey found that among the music teachers who cooperated with the survey, only one-fifth of the teachers believed that they had received psychological counseling from the school and successfully solved their own problems; nearly 60% of music teachers said that the psychological counseling provided by the school lacked pertinence and professionalism, and lacked practical solutions to their own problems. This shows that the psychological intervention strategies adopted by Chinese colleges and universities for music teachers are far from the expected results.

### 4.4. Intervention Strategies from the Perspective of Positive Psychology

#### 4.4.1. Individual Level

1. Establish a correct understanding. Correct cognition is a key factor that can ensure mental health. On the contrary, wrong cognition may lead to unhealthy psychological problems, resulting in distorted psychology. Therefore, the establishment of university teachers should establish a correct cognition, emphasizing that university teachers should examine the relationship between themselves and the teaching environment from an objective, reasonable, and comprehensive perspective, so as to build a reasonable concept and way of thinking [25]. Once the teachers have established the correct cognition, they can maintain consistency in their own and other people's eyes and gradually build a positive concept. Only in this way can they effectively control the emotional behavior behind the pressure and dissatisfaction.
2. Improve self-adjustment ability. College teachers should learn self-education on mental health and pay attention to the regulation of personal emotions. In addition, university teachers must have the ability of mental health self-education. In daily teaching life, we should teach our own psychological education methods according to our own mental state and correct self-cognitive ability. Focus on self-suggestion, self-motivation psychological hint method, timely alleviate their negative emotions, not only that but also learn to accept others, treat teachers rationally, and take a positive attitude towards their own life.

#### 4.4.2. Family Level

From the perspective of family, university teachers face the contradiction of unreasonable time allocation between work and family. In addition, it is worth mentioning that its professional characteristics determine that university teachers are a profession with high investment and low return. At present, the salary level of university teachers is generally low. It is because of these shortcomings that university teachers face specific psychological pressure. In this situation, if we still face the lack of family encouragement and support, the pressure of university teachers is unprecedented. Family members of university teachers should understand that although their material rewards are not high; they can realize the sublimation of their self-worth, so that they and their families can look at life more objectively and rationally. To sum up, as a teacher, we should feel extremely happy for the problems we are facing. This kind of happiness is inseparable from the understanding and support of the family.

#### 4.4.3. University Level

In order to strengthen the management of colleges and universities, we should reduce the research pressure on university teachers to the minimum and provide them with special rest days and comfortable teaching atmosphere, so as to alleviate the work pressure and psychological pressure of teachers. In my opinion, the more important point is to provide teachers with the opportunity and time of reeducation and learning and not only that but also to set up a special psychological consultation room for the majority of teachers and carry out teachers' psychological consultation regularly. In addition, the salary level of university teachers should be raised appropriately, so that they will not feel unfair when compared with other occupations, which can mobilize the enthusiasm of university teachers and reduce their economic burden. The research shows that colleges and universities should establish an incentive system to provide a variety of remuneration mechanisms for teachers to further enhance their work enthusiasm.

#### 4.4.4. Social Level

1. Create a good social atmosphere and improve the social status of college teachers. A perfect social atmosphere plays an important role in meeting the personalized needs of teachers, stimulating the enthusiasm of professionals, and improving the work enthusiasm of university teachers. However, the traditional sense of moral pressure has brought some moral constraints and public opinion pressure to university teachers. On the other hand, the traditional virtue of respecting teachers has been gradually weakened. First, the restriction of the society on the traditional morality of university teachers is too restrictive, which increases the psychological burden of university teachers. Therefore, this burden should be reduced. Only in this way, can we attach importance to the material and spiritual needs of university teachers to a certain extent. For example, students and parents should fully realize the hard work of university teachers and understand the good intentions of teachers for students. In order to prevent this phenomenon, the expectation of the general public for university teachers should be kept in a reasonable range.
2. Pay attention to the psychological needs of music teachers in colleges and universities and pay attention to the mental health of music teachers. The whole society has a very high social expectation for university teachers. People generally believe that university teachers have less working hours, low work pressure, and high social status, so they do not believe that the majority of teachers will have mental health problems. Obviously, this is a unilateral understanding. In fact, university teachers should be regarded as ordinary members of the society, treat them as ordinary teachers, and then get more humane care. Therefore, while paying attention to the mental health of college students, the mental health of teachers also needs to be attached great importance.

## 5. Conclusions

Studies have shown that active intervention on the mental health of music teachers can effectively reduce their occupational stress and enable them to devote themselves to work more easily and happily. The first-hand data obtained through the questionnaire survey method are of great significance for the research and proposal of countermeasures. College teachers are the focus of higher education. The psychological problems of university teachers cannot be ignored. Universities should pay attention to the psychological care of university teachers and introduce the psychological intervention mechanism. The mental health status and quality of college teachers directly or indirectly affect their own educational activities and mental health of college students. At the same time, it will also have a certain impact on other teachers. Therefore, it is very important for teachers to improve their teaching quality to enhance their self-psychological awareness and self-regulation awareness. On the other hand, both society and universities should focus on teachers' mental health and improve their psychological quality. Only in this way can the school itself and school education develop harmoniously and double win. In the following research, we will focus on the analysis of how to build a more scientific college music classroom, so as to enhance students' love and attention to the music subject, thereby enhancing the professional achievement of college music teachers.

## Figures and Tables

**Figure 1:** Physical health problems and emotional conditions.

**Figure 2:** Mental health degree of concern.

**Table 1:** Sources of stress table.

Sources of stress	Proportion (%)
Evaluation, research, and promotion of professional titles	75
Economic burden	52
Interpersonal relationship	64
Children's education	67

## Data Availability

The datasets used and/or analyzed during the current study are available from the corresponding author upon request.
